RETRACTED

# A Novel Smart City-Based Framework on Perspectives for Application of Machine Learning in Combating COVID-19

**DOI:** 10.1155/2021/5546790

**Published:** 2021-09-11

**Authors:** Absalom E. Ezugwu, Ibrahim Abaker Targio Hashem, Olaide N. Oyelade, Mubarak Almutari, Mohammed A. Al-Garadi, Idris Nasir Abdullahi, Olumuyiwa Otegbeye, Amit K. Shukla, Haruna Chiroma

**Affiliations:** ^1^School of Mathematics, Statistics and Computer Science, University of KwaZulu-Natal, King Edward Road, Pietermaritzburg Campus, Pietermaritzburg, KwaZulu-Natal 3201, South Africa; ^2^College of Computing and Informatics, Department of Computer Science, University of Sharjah, 27272 Sharjah, UAE; ^3^College of Computer Science, University of Hafr Al Batin, Saudi Arabia; ^4^Department of Biomedical Informatics, Emory University, Atlanta, USA; ^5^Department of Medical Laboratory Science, College of Medical Sciences, Ahmadu Bello University, Zaria, Nigeria; ^6^School of Computer Science and Applied Mathematics, University of the Witwatersrand, South Africa; ^7^IRISA Laboratory, ENSSAT, University of Rennes 1, France; ^8^Future Technology Research Center, National Yunlin University of Science and Technology, Taiwan

## Abstract

The spread of COVID-19 worldwide continues despite multidimensional efforts to curtail its spread and provide treatment. Efforts to contain the COVID-19 pandemic have triggered partial or full lockdowns across the globe. This paper presents a novel framework that intelligently combines machine learning models and the Internet of Things (IoT) technology specifically to combat COVID-19 in smart cities. The purpose of the study is to promote the interoperability of machine learning algorithms with IoT technology by interacting with a population and its environment to curtail the COVID-19 pandemic. Furthermore, the study also investigates and discusses some solution frameworks, which can generate, capture, store, and analyze data using machine learning algorithms. These algorithms can detect, prevent, and trace the spread of COVID-19 and provide a better understanding of the disease in smart cities. Similarly, the study outlined case studies on the application of machine learning to help fight against COVID-19 in hospitals worldwide. The framework proposed in the study is a comprehensive presentation on the major components needed to integrate the machine learning approach with other AI-based solutions. Finally, the machine learning framework presented in this study has the potential to help national healthcare systems in curtailing the COVID-19 pandemic in smart cities. In addition, the proposed framework is poised as a pointer for generating research interests that would yield outcomes capable of been integrated to form an improved framework.

RETRACTED

## 1. Introduction

The novel coronavirus named severe acute respiratory syndrome coronavirus 2 (SARS-CoV-2) has caused unprecedented numbers of deaths from coronavirus disease 2019 (COVID-19) worldwide. For instance, the United States of America recorded over 3,000 deaths within one period of 24 hours in December 2020, and the highest in the world for a single day and as of October 2020 has recorded a total of 270,642 deaths. The first human-to-human transmission of COVID-19 was reported to the World Health Organization (WHO) on 30th December 2019. Thereafter, several retrospective studies revealed that many COVID-19 patients started showing pneumonia symptoms in early December ([1–3]. Even though there are scientific controversies and theories over the date and origin of the SARS-CoV-2, it is widely accepted that the novel coronavirus originated from Wuhan, China [4]. Genomic sequences of the early isolates of SARS-CoV-2 from infected patients in Wuhan showed over 88% nucleotide homology with two bat-like SARS coronaviruses, which pointed strongly towards the zoonotic source with bats serving as reservoir hosts of the SARS-CoV-2 [4]. There are ongoing searches for possible intermediate hosts, which might have aided the transmission of the virus to humans. SARS-CoV-2 is a droplet borne pathogen that spreads by contact with humans when they are exposed to oral or nasal secretions of clinically symptomatically or asymptomatically infected persons [5].

SARS-CoV-2 has tropism in cells and tissues that express the angiotensin-converting enzyme 2 as a receptor. These receptors are mainly found in the respiratory tract and to a limited extent in the kidney, heart, and gastrointestinal tract. The virus docks onto the receptor through the receptor-binding domain (RBD) of its spike glycoprotein. This represents the first step of viral replication and pathogenesis [6]. As the virus replicates in the respiratory tract, it provokes respiratory symptoms, mainly dry cough, difficulty in breathing, and sore throat. Then, it disseminates through the blood to other tissues and organs, causing viremia and high fever. Hence, these symptoms, together with body weakness and pains, represent the primary clinical symptoms of COVID-19 [7].

The majority of SARS-CoV-2-infected persons remain asymptomatic, with the infection being self-limiting. However, some 5% of infected persons suffer severe COVID-19 [6]. The major determining factors for severe and possibly fatal COVID-19 include advanced age (>60 years) and underlying cardiovascular, immunological, metabolic, or respiratory comorbidities. Based on available scientific reports, the transmission of SARS-CoV-2 depends on human-human, animal-human, and environment-human transmission [8]. For now, preserving human life and health security is the major concern of most countries and territories. Hence, it prompted legislation to implement and enforce adequate infection prevention and control measures for these high priority pathogens [9]. Therefore, combatting the COVID-19 needs better understanding.

RETRACTED

To better understand COVID-19 in terms of its pattern of spread, identifying the most susceptible people according to their distinct genetic and physiological characteristics for COVID-19, to improve the accuracy and speed of its diagnosis, and develop new therapies, machine learning algorithms are required to analyze the large scale COVID-19 datasets [10]. As a result, scholars have attempted to apply machine learning algorithms to combating COVID-19 from various perspectives. For example, drug discovery targeting COVID-19 is proposed in Ge et al. [11]; machine learning approaches are applied in CRISPR-based COVID-19 surveillance using genomic data as proposed by Metsky, Freije, Kosoko-Thoroddsen, Sabeti, and Myhrvold [12]. Similalry, Pandey, Gautam, Bhagat, and Sethi [13] develop a system for creating awareness about the importance of hand washing to contain the spread of COVID-19, while Yan et al. [14], in their study, employed machine learning techniques to predict the survival of severely affected COVID-19 patients. More so, the classification of novel pathogens for the COVID-19 is presented in Randhawa et al. [15]; a deep learning-based system for quantifying the volume of lung infections is reported in Yan et al. [14], and automated deep learning COVID-19 patient detection and monitoring systems are reported in Gozes et al. [16], Oyelade and Ezugwu [17], and Oyelade et al. [18]; lastly, a generative network is used for the design of COVID-19 3C-like protease inhibitors [19].

However, each of these previous studies focuses on only a single aspect of combatting the COVID-19 pandemic, whereas a multifaceted approach considering all critical aspects required to fight the COVID-19 pandemic is needed. As an example, [20] reported that hospital emergency rooms across the globe experience unprecedented floods of people infected with COVID-19 needing urgent treatment. As a result, doctors have to grapple with the problem of patient's triage as they struggle to decide which of the COVID-19 patients require intensive care. For this, the condition of the patient's lungs must be assessed by doctors and nurses. However, doctors and nurses without pulmonary training cannot assess the patient lungs. At the peak of the COVID-19 crisis in Italy, doctors were faced with a serious problem of making decisions on the patient that should be given much needed assistance. Given the difficulties of making triage decisions in COVID-19 cases, a machine learning system could support doctors and nurses making clinical decisions and plays a critical role in the COVID-19 crisis by assisting hospitals in functioning better in keeping COVID-19 patients alive.

RETRACTED

A multidimensional framework for automated machine learning solutions to combat COVID-19 on different fronts could provide better means of combating the COVID-19 pandemic, for example, predicting COVID-19 vaccine immunogenicity, COVID-19 contact tracing, monitoring social distancing, and mask wearing, optimizing COVID-19 resource allocation, detecting COVID-19 severity and triage of COVID-19 patients, predicting COVID-19 patients who require a ventilator or predicting those who are beyond medical intervention, predicting COVID-19 mortality, and discovering COVID-19 drugs. All these aspects could be integrated into a single framework to work automatically within a city. Therefore, a smart city could be repurposed to combat the COVID-19 by applying a framework of multiple measures to fight the COVID-19 pandemic. Many technologies are connected to provide smart applications in smart cities, including wireless sensor networks, broadband communications services, sensor devices through the internet, and cloud services. Sullivan [21] predicted that smart cities in 2020 would be embedded with smart structures such as smart healthcare, smart security, smart mobility, smart buildings, smart governance, smart citizens, smart infrastructure, smart technology, smart energy, and smart education.

To the best of our knowledge, our proposed framework stands out from other similar existing frameworks reported in the literature; in that, this study presents the most comprehensive integration of components that are perceived to integrate well with machine learning in order to fight COVID-19 automatically across multiple dimensions in smart cities. The framework could address the unique challenges in fighting COVID-19, thereby easing the work of healthcare workers in saving lives and providing a guide for real-world execution of a program in smart cities. Yu, Wang, Liu, & Zomaya [22] pointed out that exploring such a theory is critical for providing a guide for effective applications.

The gap in literature motivating the need for this study leads to the following research questions:

- Considering the high volume and raw data generated from internet-connected sensory devices, how can machine learning models be adapted and adopted for inferring higher-level information?
- What are the challenges associated with the interoperability of internet of things (IoT) technologies with machine learning algorithms in collecting and analyzing COVID-19 data?
- Could the higher-level information be repurposed in supporting applications (such as detection, prevention, contact tracing, and alert-level dissemination systems) designed to combat the COVID-19 pandemic?
- How can a computational solution based on a robust framework be applied to evaluate the environmental and social weaknesses of a city for containing new COVID-19 outbreaks?

RETRACTED

This paper proposes a solution framework integrated with machine learning to combat COVID-19 in smart cities from multiple dimensions. The novelty of the study lies in the essential elements of the framework and how its elements such as physical structures, institutions, policymakers, medical personnel, ICT, IoT, big data, and machine learning algorithms seamlessly integrate to manage all kinds of applications and devices.

The remainder of the paper is organized as follows: Section 2 presents the background information about fundamental concepts considered in the study, Section 3 presents the proposed solution framework for combatting COVID-19 in a smart city from multiple fronts, Section 4 presents the applications of machine learning in fighting COVID-19 pandemic in smart cities, and Section 5 discusses the outcome of the study by outlining case studies on combatting COVID-19 via machine learning in smart cities, before the concluding remarks in Section 6.

## 2. Preliminaries: Overview of the Novel Coronavirus Diseases, Smart Cities, and Machine Learning

This section presents an overview of the fundamental concepts, components, and related works on which the study is focused. This general overview allows conceptualization of the proposed framework in the subsequent subsections. Our review provides details of the COVID-19 disease and its clinical manifestation and also of the concept of smart cities as they relate to IoT. In addition, the background to machine learning and its associated algorithms is discussed.

### 2.1. Novel Coronavirus Disease: Background and Primary Clinical Features

In this subsection, an attempt is made to present fundamental knowledge about the disease COVID-19 caused by the novel coronavirus SARS-CoV-2, with background information and clinical features which are relevant for the implementation of the proposed framework.

#### 2.1.1. Background of Novel Coronavirus SARS-CoV-2 and COVID-19 Disease

Out of the seven known coronaviruses, SARS-CoV-2 is the third-most highly pathogenic coronaviruses to have afflicted the human race. As the SARS-CoV-2, the etiological agent of COVID-19 spreads across more than 210 countries and territories, infections, and subsequent fatality rates continue to rise. Accordingly, several preventive and control measures have been adopted to halt the spread of the SARS-CoV-2 and minimize COVID-19-associated death. As of 7 : 30 AM GMT+1, 27^th^ April 2020, there were over 3 million confirmed cases of SARS-CoV-2 infection globally with a case fatality rate (CFR) of around 7.0% (Worldometer, 2020). At that time, European and American countries, with only a few Asian countries, appeared to have the worst CFRs associated with COVID-19, with the least being in Africa, without any categorical explanation for this variation. Several observers have attributed the low incidence rate of COVID-19 in sub-Saharan Africa to underdiagnosis, probably due to inadequate molecular diagnostic capacity, but variation in the genetics, strains, viral protein mutations, and host immune response could have contributed to SARS-CoV-2 virulence and pathogenesis [23].

RETRACTED

Although there have been controversies about the origin of SARS-CoV-2, several studies have traced the zoonotic source of this virus to the first patients exposed in a live animal market in Wuhan, China [4]. Subsequently, efforts have been made to search for a reservoir host and intermediate hosts of SARS-CoV-2, from which the infection might have spread to humans. Initially, two snake species were identified in this regard. However, the only consistently identified SARS-CoV-2 reservoirs have been mammals such as bats [4, 24]. In particular, early isolates of SARS-CoV-2 from infected patients in Wuhan showed genomic sequencing of some SARS-CoV-2 isolates to have 88% nucleotide homology with two bat-derived SARS-like coronaviruses [25], thus indicating bats as the most likely reservoir hosts for SARS-CoV-2 [25].

The first principal transmission mode of the SARS-Co-V-2 is through droplets emanating from the respiratory system of infected people. These droplets are transferred by coughing and sneezing so that when they come into contact with the respiratory system of uninfected persons, it may cause a COVID-19 infection. These, therefore, form the second principal transmission mode, which is by contact [26]. Although younger persons have exhibited some resistance to the disease due to their strong immune systems, studies have shown that people of all ages are at risk of contracting it. The aged who have had contact with infected persons or surfaces carrying the virus often progress quickly to acute respiratory distress syndrome (ARDS) and multiple organ failures. Infected younger persons may succumb to mild syndromes like fever, fatigue, and dry cough, with only a small percentage of cases degenerating quickly, as seen in the elderly. The disease's propagation level in a city or population is often evaluated using fatality rates and reproduction number (popularly referred to as R_0_ value, see Section 2.1.2) and, recently, the index c value [27]. The effect of this propagation has spilled over into social economic problems, which are directly a result of contracting the GDP growth of countries due to lockdown enforced in several countries [28].

RETRACTED

#### 2.1.2. Clinical Features of Novel SARS-CoV-2 and COVID-19 Disease

Virologically, SARS-CoV-2 is a single-stranded RNA virus with positive polarity and variable open reading frames (ORFs) [29]. It has been shown that two thirds of the SARS-CoV-2 genome is located within the first ORF, which translates the pp1a and pp1ab polyproteins. These polyproteins encode 16 nonstructural proteins [29], which are the remaining ORFs code viral structural and accessory proteins of SARS-CoV-2. The remaining one third of the genome codes the nucleocapsid (N) protein, spike (S) glycoprotein, matrix (M) protein, and small envelope (E) protein of SARS-CoV-2. Of these four proteins, the S glycoprotein is key because it plays a role in attachment to host cells and the pathogenesis of COVID-19. This protein, alongside the viral RNA-dependent RNA polymerase (RdRP), has largely been utilized in the synthesis of primers and antigens for, respectively, molecular and serological tests of SARS-CoV-2 infection [30].

RNA viruses, including SAR-CoV-2, have high mutation rates, which is significantly correlated with enhanced virulence and evolvability [31]. At the proteomic level, amino acid substitutions have been reported in the NSP2, NSP3, and S proteins [32]. Another study of interest has suggested that NSP2 and NSP3 mutations play a significant role in the virulence and differentiation mechanism of SARS-CoV-2 [33]. Of interest is the mutation in S-protein. This has made scientists explore the possible differences between the host tropism and the transmission rate of SARS-CoV-2. It is worth noting that the NSP2 and NSP3 mutations in SARS-CoV-2 were isolated from many COVID-19 patients in China [33]. These have mutations sparked scientific interest in genomic surveillance of SARS-CoV-2 to determine the correlation between these mutations and virulence diversity, with its implications for reinfection, immunity, and vaccine development [34].

A measure of the transmissibility or infection rate of SARS-CoV-2 can be measured by *R*_0_, which predicts the number of people to whom an infected person could transmit SARS-CoV-2 in a population with no prior immunity to the pathogen. Generally, the higher the *R*_0_, the more contagious the pathogen. An *R*_0_ of <1 means that the outbreak would die out, while *R*_0_ > 1 means the infection will continue to spread [35]. Based on available genetic analysis, SARS-CoV-2 is related to SARS-CoV-1, which along with MERS-CoV, is endemic in certain countries; so, *R*_0_ is not very high. However, an early report on mathematical modelling for SARS-CoV-2 revealed an *R*_0_ of 2 to 3 [14], which could explain why SARS-CoV-2 is more contagious than either SARS-CoV-1 or MERS-CoV. This model highlights that a single SARS-CoV-2-infected individual has the ability to infect two to three uninfected persons [36].

RETRACTED

Infection by SARS-CoV-1 occurs through contact with respiratory droplets, which are the size of nanoparticles and can contaminate surfaces and hands, and where they remain stable for hours [36]. Hands, therefore, become a mechanical vector and are, thus, a potential site to eliminate the virus and prevent it from invading the body. However, suppose the virus is not eliminated at this stage, in that case, it can move towards its predilection site (i.e., cells of the lungs), where it attaches using its spikes and uses the angiotensin-converting enzyme-2 (ACE-2) as receptors to gain access to epithelial cells of the respiratory tract. At this stage, SARS-CoV-2 compromises innate lung immunity [36]. It then takes advantage of these cells as a replication site. The virus regenerates and sheds by disassembling itself and utilizing the machinery of the alveoli cells, to be precise, the Golgi apparatus, to reproduce, and repackage itself [36].

The SARS-CoV-2 exists so that it can replicate and disrupt the protective function of the ACE-2 receptor, which induces the process of fibrosis (scarring). It has been shown that patients with fatalities associated with SARS-CoV-2 present a characteristic ground glass effect in their lungs, and this sequela impedes efficient oxygenation. As the body tries to compensate for this deficiency, the result is a severe acute respiratory syndrome (SARS), in which it becomes impossible for the respiratory system to make oxygen available to the rest of the body (hypoxia) [36]. This ultimately results in multiple organ failures. Based on available clinical data, those susceptible to developing a severe form of SARS-CoV-2 infection include the elderly (>60 years) and persons with underlying disease conditions (e.g., cardiovascular, metabolic, respiratory, and immunological disorders) [37].

When susceptible individuals get infected by SARS-CoV-2, that person may either remain asymptomatic (no apparent illness) or be symptomatic. If symptomatic, the disease passes through three stages of severity. Patients present with mild clinical symptoms in the early infection stage (Stage I), including dry cough, diarrhea, fever, and headache. This could last for 3 to 5 days. This stage is usually accompanied by lymphopenia (low white blood cell counts), elevated prothrombin time, D-dimer, and a mild increase in lactose dehydrogenase (LDH). Almost all (98%) of SARS-CoV-2-infected patients remain at this stage and eventually recover. However, those with underlying medical disorders may proceed to stage II (Pulmonary Phase), predominantly characterized by shortness of breath and hypoxia (inadequate oxygen supply to the body), which could last from 5 days to 3 weeks. At this stage, patients would display an abnormal chest radiograph, transaminitis, and declined procalcitonin levels. Very few patients (2%) proceed to this severe stage of COVID-19. Stage II (hyper-inflammation phase) is largely characterized by acute respiratory distress syndrome (ARDS), severe inflammatory response syndrome (SIRS), shock, and cardiac failure. The majority of patients who reach this stage eventually die. At this stage, COVID-19 patients experience significantly high blood inflammatory markers such as elevated C-reactive protein (CRP), interleukin-6 (IL-6), D-dimer, and ferritin. In addition, affected patients present with the increased blood level of cardiac markers, especially troponin and N-terminal (NT)-prohormone B-type natriuretic peptide (NT-proBNP) [38].

RETRACTED

Diagnostically, the use of viral culture for establishing acute COVID-19 diagnosis is not practicable due to the long turnaround time (3 days) for SARS-CoV-2 to cause obvious cytopathic effects (CPE) on Vero E6 cells. In addition, isolation of SARS-CoV-2 is laborious and requires biosafety level-3 (BSL-3) facilities, which are unavailable in most healthcare centers, especially in developing countries. So far, all available serum antigens (such as the S-glycoprotein) and antibody (IgA, IgM, and IgG) detection tests have not been validated by the WHO. However, it has been suggested that serological assays could assist in analyzing an ongoing SARS-CoV-2 outbreak and retrospective evaluation of the incidence rate of an outbreak [9]. In some instances, where epidemiological data of suspected cases correlates to SARS-CoV-2 infection, the demonstration of fourfold rising antibody titer between acute and convalescent-phase sera could support the diagnosis of COVID-19 when RT-PCR results are negative [9]. In addition, it has been revealed that a significant proportion of COVID-19 patients have tested RT-PCR negative despite having suitable clinical features and radiologic findings that are highly indicative of SARS-CoV-2 infection [39]. In most cases, these are termed false negatives, which could have been due to wrong sampling if SARS-CoV-2 had been present in the lower respiratory tracts rather than in the upper respiratory samples usually collected for laboratory diagnosis. Hence, this difficulty in diagnosis poses a challenge in the proper evaluation of SARS-CoV-2 symptomatic patients [40].

RETRACTED

### 2.2. Rudiments of Smart Cities and Machine Learning

In this section, the discussion of the concept of a smart city, including case studies and the brief explanation of machine learning, is intended to help readers new to these domains comprehend the concepts of smart city and machine learning.

#### 2.2.1. Smart Cities

There is, as yet, no universally accepted standard definition of a “smart city.” However, a smart city may be understood as a city that encourages the prudent utilization of quality resource management and the provision of services within a limited time. Information and communication technology (ICT) is one of the major components and an integral element in innovative city projects. The operations in a smart city cannot be achieved with ICT in isolation. This state-of-the-art view of city development has resulted in the new smart city model. The quality and scale of cities have grown significantly as a result of urbanization since the industrial revolution. The expansion in urbanization has prompted many challenges, including [41]

- Large scale consumption of resources
- The degradation of the environment
- The unfair widening of the gap between the rich and the poor

The smart city model can help cities achieve sustainability goals, such as high-level efficiency, high economy, an improved standard of living for people, and a beautiful city environment. Many criteria to assess the smartness of a city have been proposed, which include all or some of the following: smart energy production and conservation, smart mobility, smart economy, smart living, ICT economics, smart environment, smart governance, and the connection between the standard of living and smart society [41]. To put a smart city in its proper position, a smart city is the combination of a wide range of services that are required by a city and the need to offer the services in a way that complies with the current administration requirement through the use of state-of-the-art technology.

#### 2.2.2. Case Studies of Smart Cities

To buttress our contention about the potential for smart cities in providing critical support to their population, we briefly review three case studies of the application of IoT technology to a city, namely, Kuala Lumpur, Copenhagen, and Stockholm.

*(1) Case Study 1: Kuala Lumpur, Malaysia*. In Kuala Lumpur, many projects in relation to a smart city are designed to use the city's resources optimally. For instance, many innovations have been implemented in the transport sector to reduce traffic congestion. The innovations include using smartphones for flight check-in, train and bus schedules being monitored through electronic boards in the city train and bus stations, and smart cards, referred to as “touch and go,” and are commonly used to avoid long queues in purchasing bus or train tickets; an application referred to as “GrabCar” is used to book a cap and track its position and the estimated time of arrival to the pick-up position. The weather can be monitored through smartphones, such as showing the daily temperature in different city locations. Nonsmoking areas are also embedded with sensors to trigger an alarm in case of smoking cigarettes in the nonsmoking zone. In addition, many of the vehicles in Kuala Lumpur are hybrid, which enables switching the engine from electric to petrol and back to electric, as needed.

*(2) Case Study 2: Copenhagen, Denmark*. The Boyd Cohen list of smart cities in Europe ranked Copenhagen in eighth place [42]. For Copenhagen, numerous smart city projects were analyzed from the perspectives of success factors and economics. Copenhagen has the vision of becoming the world pioneer carbon-neutral capital by the year 2025. As such, Copenhagen is presently implementing innovations in the field of transportation, waste management, water supply, heating, and sources of alternative energy to support the 2025 target vision for the city and enhance sustainability. Copenhagen has currently expanded its network of cycle lanes to be embedded in the broad transportation concept to improve traffic flow in the city (Catriona [43]).

RETRACTED

### 2.3. Machine Learning

Machine learning is a field of science that centers on how a computer learns from data [44]. According to Portugal, Alencar, & Cowan [45], machine learning is an algorithm that “uses computers to simulate human learning and allows computers to identify and acquire knowledge from the real world, and improve the performance of some tasks based on this new knowledge.” Machine learning is a subdiscipline in artificial intelligence and cuts across many fields of studies that correlate with data mining, pattern recognition, computer science (theoretical), and statistics [46]. In statistics, it seeks to determine the relationship that exists in data, whereas in computer science, it emphasizes the effectiveness of the computational algorithm. Machine learning research in computer science examines the algorithm used for the learning to make a prediction based on data. To achieve that, the input data is employed to construct a model so that a data-driven decision can be made with various static program instructions [47]. Machine learning algorithms can be broadly categorized into supervised learning, unsupervised learning, and semisupervised learning.

Supervised learning (input observation mapped with output observation) is learning where the input observation consists of features, and the output observation consists of labels [48]. Thus, it constructs a model by utilizing a labeled dataset as input [49] and produces labeled output data. The primary purpose of supervised learning is to drive a functional correlation from the training data with well-generalized testing data. Some examples of supervised learning algorithms are employed in classification and regression problems, including naïve Bayes, decision tree, and logistic regression. On the other hand, unsupervised learning is a learning algorithm that is employed when there are difficulties in finding the labeled sample, since it does not rely on previous training for mining the data. The primary purpose of unsupervised learning is to find a correlation between the samples behind the observation. One of the notable examples of unsupervised learning is a clustering system. Semisupervised learning is a combination of supervised and unsupervised learning, which uses a small amount of labeled data and a huge amount of unlabeled data [50] during the training process. Information recommendation systems and semisupervised classification are examples of a semisupervised learning algorithm.

The machine (and deep) learning algorithm can be applied in many research fields, including natural language processing [17], medical diagnosis, financial data analysis, bioinformatics, and video surveillance. The following section presents our approach to harmonizing machine learning algorithms and IoT technologies using a novel framework. Furthermore, a detailed discussion on the applicability of the proposed framework in combating the COVID-19 pandemic is presented in Section 4.

## 3. Proposed Method

The ubiquitous nature of internet-connected sensory devices, which are often capable of generating relevant data for analytics purposes, has motivated the approach promoted in this study. These devices can capture a high volume of structured and unstructured data based on the time and location of the physical world. We argue that intelligently processing these volumes of data requires learnable algorithms that, with minimal human intervention, can derive a pattern sufficient to present higher-level information to support combating COVID-19. Hence, this section presents a novel framework that intelligently allows for the interoperability of IoT concepts and machine learning models.

RETRACTED

### 3.1. The Smart City-Based Machine Learning Framework for Combating COVID-19

To address the multiple dimensional challenges posed by the COVID-19 pandemic, as outlined in Section 1, we propose that a framework is required within the smart city context to allow decision makers to make the crucial decisions on the best ways to combat COVID-19 from multiple dimensions. The framework consists of multiple components, as shown in Figure 1. Each component has a major impact on enhancing the quality of the analytics to combat COVID-19.

### 3.2. Modules of the Smart City Framework

The smart city-based framework has four core modules, namely, smart city environment, image and clinical collection strategy, image preprocessing and analytics, machine learning models, cloud-based storage, and evaluation strategies. The following subsections provide details of the modules.

#### 3.2.1. Smart Environment

Smart city technologies have recently demonstrated their potential for enhancing citizens' quality of life. Many smart-based technologies have arisen from the adoption of the internet of things (IoT), which has led to the development of intelligent applications such as smart homes, smart grids, smart transportation, smart industry, and smart healthcare. Moreover, recently sensors and video cameras surveillance have become part of smart city monitoring; they can also be used for early detection of a pandemic. During the COVID-19 pandemic, smart technologies could help in tackling the major clinical, social, and economic problems due to the disease. Specifically, health agencies may utilize IoT platforms to access data for monitoring the COVID-19 pandemic. For example, “Worldometer” allows viewing of instant updates about the severity of COVID-19 for the entire world. These updates include daily new cases and deaths due to COVID-19, cumulative numbers of cases and deaths, and distribution of COVID-19 by country [51]. In Figure 1, we demonstrate a smart environment that could be used for healthcare purposes, in which the IoT and various sensors and monitoring devices interact within a limited area to generate data on clinical signs and symptoms. These devices are connected via next-generation wireless connectivity, which can efficiently transfer the collected data to be stored in a big data lake. Big data plays a critical role in smart cities because its ecosystem of data analytics can allow decision makers to decide critically on the best strategy to be developed to combat COVID-19. With big data and with adequate smart city framework implementation, users can be traced at all times with the potential to mitigate any health problems they might encounter during their movement. Therefore, improving the efficiency and effectiveness of a smart city framework would, in turn, improve the lives of the citizens in the smart cities. A literature review was conducted by Al-Turjman [52], which presents comprehensive background about 5G standards and their specific applications for the IoT and an overview of recent developments in use of smartphone sensors that could contribute to a scalable operation in smart social spaces.

RETRACTED

#### 3.2.2. Image and Clinical Data Collection Strategy

The image and clinical data generated in real-time for smart cities can be subjected to big data processing to understand healthcare trends, model risk associations, and predict outcomes. The government authorities can use the results of the big data lake with private/public healthcare providers to improve healthcare services to the citizens; this process would continue until the government and healthcare services providers satisfy the citizens living in the smart cities. The various means of collecting data on a large scale include social media platforms such as Facebook, Twitter, Google+, Instagram, healthcare services data collected during diagnosis and treatment, and tracking of monitoring devices such as GPS and vehicle tracking systems, smartwatches, and sensors. All collected data would be integrated and stored in a single location within the smart city to be accessed by the authorized entities. The technologies that make storage of such dad possible are Hadoop distributed file system (HDFS) and NoSQL, in which both structured and unstructured data can be stored and processed. Balduini et al. [53] proposed a new conceptual framework that uses a variation of big data sources. The unified approach in their framework uses spatial and temporal analysis on a heterogeneous stream of data. Their results show the proposed framework's generality, feasibility, and effectiveness across many cases and examples obtained from real-world requirements using data collected in many cities.

#### 3.2.3. Preprocessing

In order to provide more accurate and better input to achieve more reliable results in the detection and prevention of COVID-19 cases, data preprocessing is considered an important first stage. The first step in preprocessing is to extract all the relevant COVID-19 data from storage. The second step is to perform data fusion, whereby the collected data are integrated to produce more consistent, accurate, and useful information. The third step during preprocessing of COVID-19 data is to reduce dimensionality, in which the number of variables is reduced by extracting a set of main variables. The fourth and fifth steps focus on feature extraction and selection. The last two steps are very important in filtering irrelevant or redundant features from the selected datasets. The last step involves a basic statistical analysis of COVID-19 data in order to interpret the data before intelligence-based algorithms are applied.

RETRACTED

#### 3.2.4. Analytics

Recently, image processing in healthcare using convolutional neural networks has become a significant approach for handling large quantities of images generated from smart cities. Allam and Jones [54] discuss the universal data sharing standards that are coupled with AI to benefit urban health monitoring and management. Our proposed framework can incorporate various machine learning and deep learning algorithms to develop the analytical model. These algorithms range from traditional shallow approaches such as neural networks, decision tree, naïve Bayes, and *K*-nearest neighbor. These algorithms can be applied to run on COVID-19, a dataset in applications that help combat COVID-19 in hospitals, in smart cities, and across the world. These applications include detecting and preventing the spread of COVID-19, forecasting the next epidemic, diagnosis of cases, monitoring COVID-19 patients, tracking potential patients, suggesting methods for vaccine development, helping in COVID-19 drug discovery, and together providing a better understanding of the effect of the COVID-19 virus in smart cities.

*(1) Social Media Information Verification*. The COVID-19 pandemic has brought associated challenges of fake news, including conspiracy theories. Since the COVID-19 pandemic started, there has much fake news regarding its origin, cures, mode of spread, treatment, and many other myths. This is especially prevalent on social media platforms such as Facebook, Twitter, Instagram, and YouTube. In a smart city, citizens would voice their opinions on social media regarding COVID-19 to generate unstructured data. It is reported by Obeidat [55] that no systematic quantitative study has been conducted to ascertain the magnitude of the problem of myths perpetuated on social media around COVID-19, but certainly, the figures for misinformation about COVID-19 are significant. The fake news regarding COVID-19 can come in the form of manipulated content, misleading content, satire, false context, malicious accounts, fabricated content, false connections, and imposter content. Therefore, machine learning or deep learning algorithms can be applied to detect fake news regarding COVID-19 on social media and alert citizens living in smart cities.

*(2) Prediction of Future Pandemic*. Although being the worst pandemic in recent times, this pandemic has, nevertheless, come in the time of the digital age. Therefore, every aspect of the analysis can now be captured, including at a macrolevel, logistically, and biologically, in terms of data; this will definitely be fruitful for predicting the behavior of this new pandemic or of unknown future pandemics. For example, with the help of the machine learning approach (random forest), Eng, Tong, & Tan [56] could predict possible zoonotic strains of influenza, i.e., some viruses that usually only affected animals but might also be dangerous to humans. This, therefore, implies that machine learning could help to predict future pandemics arising from any species. The only limitation is that the data could be from a different domain, e.g., the source of COVID-19 is possibly from “bats;”,so, pandemic sources may be different from those encountered in the past (for instance, having a different genome structure, etc.). Further, traditional machine learning requires the data distribution to be from the same domains in training and testing. However, transfer learning (TL)—a type of machine learning—can effectively handle situations where training and testing data might be from different data distributions. That is, the knowledge learned from the past pandemics could be used in future situations with a new domain, even with smaller amounts of data. Such a scenario is shown in Figure 2, where the pretrained model from the current COVID-19 pandemic (with large data and labels) could be used, with significantly less data and labels, to predict future pandemics, prepare the smart city for that situation, and quickly help address the spread of the disease.

RETRACTED

The modules of the smart city-based framework for combating COVID-19 shown in Figure 2 present very promising applicability; this study further provides a perspective on how this is achievable. The following section is focused on detailing this aspect.

## 4. Perspective on the Applicability of the Proposed Framework

As an interconnected urban society, the smart city implies collecting data every moment from several embedded devices, which means that smart cities can work effectively with machine learning approaches during this COVID-19 pandemic. Machine learning techniques are dependent on data for better learning and predictive models, through which they can bring out some intrinsic and valuable insights to help the decision makers in smart cities take preventive measures during the COVID-19 pandemic. Different machine learning techniques operate with other fields of artificial intelligence (AI), which gives the model its ability to provide a rich self-learning platform. It is important to discuss the role of AI and machine learning in combatting COVID-19, because the data availability is limited, and we have to deal with real-time data streaming. Thus, the significance of self-learning systems becomes much more desirable in smart cities.  Figure 3 demonstrates the overall flow of how AI and machine learning approaches can help in fighting the COVID-19 pandemic in smart cities.

RETRACTED

As shown in Figure 3, several types of data are generated from the information and communication technology equipment embedded in smart cities. These are as follows:

- The statistical data that usually contains the cumulative daily number of identified cases, number of new positive cases, number of deaths, number of recovered cases, etc. would help predict future cases to prepare for emergencies
- The epidemiological data primarily concerns all the clinical patient test data, data relating to tests on different medications, various drug trials, patients' medical histories, patients' responses to different medications, etc.
- The real-time surveillance data generated from sensors and cameras in the smart cities would also be helpful to track and prevent the spread of COVID-19. For example, one of the initial identifiers of COVID-19 is based on symptoms of fever; so, body temperature from facial recognition and other personal information can be monitored

The data is processed and analyzed through machine learning approaches for extracting insights in various applications. The applications of machine learning in different aspects for combatting COVID-19 are discussed in the following subsections.

### 4.1. Prevention and Precaution

Based on the statistical data, the machine learning model can be used to predict the nature of the identified cases to take better preventive measures. During the situation of a pandemic, there may be a degree of chaos. The requirement for rapid and large-scale testing of individuals is very challenging. So, rather than going door to door to each patient, a faster approach would be more acceptable, even if less accurate. Machine learning may help in quickly diagnosing the patients in the smart cities as follows:

- Facial recognition with the help of sensors and cameras to scan the patients for body temperature and personal information so that if the particular patient is positive, then their nearby individuals can be tested and alerted to their status
- Helping patients get information and create self-awareness with the AI-powered chatbots because the medical professional might find it impossible to address these queries during the COVID-19 pandemic because of the exceptionally high number of patients they must help
- Using the data from smartphones and wearable smartwatches to monitor the citizens' heart rate and daily activity

Although predictions based on the statistical data may not be 100% accurate, they can nevertheless enable the decision makers in smart cities to institute some preventive and proactive measures.

RETRACTED

### 4.2. Prediction Models

Medical science (especially dermatology) was one of the real-world fields where AI and machine learning approaches were successfully implemented. Computer vision and machine learning prediction models can identify patients' most common dermatological diseases simply by learning from images. In the case of COVID-19, based on some set of crucial features (set of symptoms), machine learning approaches can help in identifying and predicting the following:

- A person infected with COVID-19
- A positively diagnosed COVID-19 patient who needs to be hospitalized
- According to the range of treatments available, the chances of a COVID-19 patient being successfully cured or dying

Pourhomayoun and Shakibi [57] used machine learning techniques to predict the mortality rate of patients affected by COVID-19. They used machine learning algorithms such as random forest, logistic regression, decision tree, support vector machines, and artificial neural networks to give up to 93% total accuracy in predicting the mortality rate. Moreover, the study also used machine learning models to extract the essential and unique symptoms and features to detect the virus.

#### 4.2.1. Prediction of COVID-19 Pandemic

Different studies have been conducted to predict the likely occurrence of the COVID-19 pandemic [58]. For instance, Ndiaye, Tendeng, and Seck [59] conducted a global prediction study on the COVID-19 pandemic between January and April 2020. The study employed prophet [60], a tool for predicting time series data; it depends on the additive model that fits real nonlinear trends with daily, weekly, and annual seasonality and holiday effects. Four countries of Italy, China, Senegal, and Iran were selected as case studies for the research. However, the predictive performance of the study showed that the COVID-19 pandemic in countries like China could be optimistically estimated to end in a few weeks. In another perspective, Wang and Wong [26] proposed COVID-Net, which uses a convolutional neural network design to identify COVID-19 cases from chest X-ray (CXR) images. The study utilized the CXR dataset, which comprised 13,800 chest radiography images obtained from 13,725 patients from three public datasets. The experimental analysis shows that the proposed COVID-Net attained a predictive accuracy of 92.6% on the test data, indicating the importance of combining human and machine collaboratively in the design strategy for building modified deep neural network architectures faster fitted around the data, task and working requirements. In another study, Yang et al. [61] proposed a modified susceptible, exposed infections removed (SEIR) model and AI prediction of COVID-19 pandemics. The study employed the most up to date COVID-19 epidemiological data together with population migration data obtained prior to and after 23rd January 2020 into the SEIR model. In addition, a machine learning approach was employed to train on the 2003 SARS data for the pandemic prediction. The predictive result of the study shows that the pandemic of China was expected to be at peak by late February and then show a gradual decline by the end of April. However, the COVID-19 cases would have risen higher than expected in mainland China should the implementation of the proposed model have been delayed for as little as five days.

RETRACTED

In their study on the outbreak of COVID-19, Gozes et al. [16] developed an artificial intelligence-based automated computer tomography (CT) image analysis tool using a deep learning approach for the detection, tracking, and quantification of COVID-19, which could distinguish patients infected with COVID-19 and those who were not. The study utilized various global datasets, which included those for Chinese disease-infected areas. Various retrospective deep learning experiments were performed to analyze the system performance in identifying speculated thoracic computer tomography features of the COVID-19 for the evaluation of disease evolution in each patient. One hundred and fifty-seven (157) patients were selected from the US and China for the testing sets. The model's classification performance attained 0.996% AUC, 92.2% specificity, and 98.2% sensitivity on Chinese control and infected patient datasets. This shows that the proposed model could attain high predictive performance in identifying, tracking, and quantifying the COVID-19 cases. Similarly, Narin, Kaya, and Pamuk [62], in their proposal for automatic prediction of COVID-19, employed a deep convolutional neural network built on chest X-ray image and a pretrained transfer model that includes the InceptionV3, Inception-ResNetV2, and ResNet50 models to attain higher predictive performance with a small size of X-ray dataset. The experimental results attained an optimum result of 98% accuracy on the ResNet50 pretrained model among the three selected models. The research results show that the model can assist doctors with decision-making in clinical practice as it uses transfer learning to detect the early stage of COVID-19 in infected patients.

RETRACTED

#### 4.2.2. Forecasting of Mortality

Since the outbreak of the COVID-19 pandemic in Wuhan city, China, in December 2019 to the time of the study, the number of confirmed deaths has risen to over 115,000, which indicates a weekly doubling of the number of deaths [63]. There appear to have been discrepancies between the mortality statistics and reported cases, which may have resulted from test policies. Thus, the daily report of deaths on COVID-19 has been at variance with the actual deaths over time. Accurate death rate estimation is important as it is a key factor in deciding whether a highly infectious disease should be a public concern. Consequently, there is a need for reliable estimates of numbers for mortality from COVID-19, the date for the peak of deaths, and the period of highest mortality, which all assist decision makers in responding to the present and future pandemics.

A statistical model, known as Global-19, was developed by Brown et al. [63], which gives an estimate of mortality trends between 12th April 2020 and 1st October 2020 for 12 countries (USA, China (Hubei), Italy, Spain, France, UK, Belgium, Iran, Netherlands, Germany, Canada, and Switzerland). The mortality data were collected from the WHO daily reports for each country and some other online data. Similarly, Wang et al. [26] employed the patient information-based algorithm (PIBA) to determine the mortality rate for the COVID-19 pandemic in real-time with forecasts of future deaths. The data was collected from three public sites for COVID-19 patients in Wuhan, China. The data consisted of daily numbers of patients newly infected with COVID-19, the patients that had died of the infection, the patients in a critical condition who had been admitted to an intensive care unit (ICU), and people who had been in close contact with the source of infection. The findings show that the average time between the beginning of the infection to the time of death was 13 days. This prediction is based on the data collected from Wuhan, which was the first city with confirmed records of deaths related to the COVID-19 pandemic.

### 4.3. Resource Allocation

Resources required to manage the COVID-19 pandemic become scarce due to the very high number of people needing them. These resources include ventilators, masks, testing kits, personal protection equipment, and sanitizers. The problem of resource allocation is an NP-Hard problem, and it is impossible to solve in a polynomial time. Considering the urgency of the emergency created by the COVID-19 pandemic, machine learning can be very beneficial in predicting the best allocation of resources using linear and logistic regression. The machine learning model may provide feasibility and close to optimal resource allocation even on a small training dataset (as is the case for COVID-19).

RETRACTED

### 4.4. Vaccine Development

The process of discovering a new vaccine based on the available clinical data could take a long time. But with the help of machine learning approaches, the overall process can be reduced significantly without sacrificing the quality of the vaccine. For example, Ekins et al. [64] report on the use of the Bayesian machine learning model in a study to develop a vaccine for Ebola. Also, Zhang et al. [65] also used the random forest algorithm to improve the accuracy of the scores while working on the H7N9 virus. Currently, there is much effort in the scientific community applying machine learning to search for a design for the COVID-19 vaccine. Gonzalez-Dias et al. [66] reported on the stages of using machine learning to predict vaccine immunogenicity and reactogenicity signatures. The stages involve data preparation, vaccines, and relevant gene selection, selecting the suitable machine learning algorithm for modeling and performance evaluation of the predictive model.

### 4.5. Drug Discovery for COVID-19

Since the start of the COVID-19 pandemic, it has become necessary to identify drugs that can be employed to treat the disease. In this regard, machine learning can help identify existing drugs that may be effective in treating COVID-19. Machine learning can learn from drug and protein structures and predict their interaction to warrant clinical studies. Various approaches have been used to find the right drugs, either by repurposing existing ones (therapeutic) or discovering a new one. The application of machine learning and the development of the new models have made researchers focus on the application of machine and deep learning models to discover drugs that could bring a cure for COVID-19. A review of some of the studies that applied the machine or deep learning approach for drug discovery and vaccine for COVID-19 is summarized in Table 1.

## 5. Results and Discussion

In this section, we present the study's findings and reinforce the importance of the proposed framework by illustrating its use in cases where machine learning techniques are applied to help in combating COVID-19 in smart cities.

The key outcome of this study is the proposed framework and its wide-ranging applicability to the advancement of global efforts in curbing the devastating effects of COVID-19. The findings from this study have showed that handcrafted and manually driven mechanisms for managing COVID-19 remain ineffective as the outbreak has been overwhelming, defying such mechanisms. The pervasive nature of data-driven smart devices and applications continue to provide an intelligent and scalable solution for achieving a secure city in the event of local epidemics or global pandemics such as COVID-19. This finding is further supported by Shorfuzzaman et al. [69], who argued that mass video surveillance has great potential for managing social distancing as a panacea for propagating the disease. Their study echoes the aim of this study, which is to demonstrate that data-driven driven machine learning frameworks, dependent or sensory devices, will allow for their artificial deployment in smart cities for curbing COVID-19. This study has also shown that, in addition to the benefit of managing social distancing through surveillance, such video files could also provide contact tracing applications with input in chronicling events and persons needing tracing. Confirming the methods used in this study and its findings concerning the profitability of machine learning to cities overwhelmed by COVID-19, another related study by Allam et al. [70] noted that 6G technology, including digital twins and immersive realities (XR) would support the socioeconomic position of its population.

RETRACTED

Countries across the globe have had their share of first, second, and even third waves of the pandemic and are beginning to look towards a postpandemic era with the digitalization of the city system to manage a future outbreak. Again, this concretizes the critique presented in this study, highlighting the need to “smart up” the systems that drive cities. The study of Graziano et al. [71] supports the potency of the framework proposed in this study. The authors noted that governments are now considering a more inclusive techled urban development, in other words, smart cities. We argue that in developing such a techurban settlement, the outcome of this study presents authorities with a machine learning-driven framework for curtailing and managing any subsequent waves of the disease. For instance, in leveraging the real-time data collection through sensory devices in smart cities, studies using machine and deep learning algorithms have built temporal learning algorithms. Sun et al. [72] have supported this claim by applying deep learning, a submodel of the machine learning model, in projecting the level of COVID-19 disease outbreak using temporal data that are richly generated in a smart city such as that driven by our proposed framework. On the imaging and preprocessing case proposed by the framework in this study, Lassau et al. [73] showed that by intelligently integrating the performance of deep learning models with related variables (e.g. both clinical and biological), the severity of the disease in patients can be predicted ahead of time. Again, the adoption of the framework proposed in this study presents city officials with a potent tool for managing future events. Furthermore, the works of Shorten et al. [74] and Pan et al. [75] demonstrate the importance of integrating machine learning algorithms in the city-wide management of COVID-19, as can be achieved by adopting the framework proposed in this study.

RETRACTED

The user cases discussed below can help readers understand exactly how machine learning could assist in fighting the COVID-19 pandemic. As such, other nations can share their expertise in fighting the COVID-19 by applying the machine learning approaches.

### 5.1. Case Study: New York City

In New York City, there are heavy numbers of cases of COVID-19 patients and those exhibiting the symptoms. The medical staff in New York hospitals is overwhelmed by the extremely high numbers of COVID-19 patients. As a result, the medical staffs face difficulties in deciding which of the COVID-19 patients requires emergency treatment and which patients might be beyond medical intervention. To speed up such decision making for the medical staff in New York hospitals, a machine learning system has been developed through training of the system to provide clinical decisions that support the triage of patients. This system is now used in hospitals to assist with clinical decisions [20].

### 5.2. Case Study: China

China is well known for the massive amount of data generated from its citizens. China installed a network of over 200 million surveillance cameras across the country. In addition to these video surveillance cameras, biometric scanners were installed in the doorways of residential complexes. As a form of registration, any resident or person that is leaving the residential building must present his or her face to the biometric scanner. After that, the embedded intelligent systems process the data and track the person location through video surveillance. All the information is stored in a central database in which the machine learning algorithms run the data to determine the possible social interactions of the person when they leave the residential building [76].

### 5.3. Case Study: Canada

Human movement across the globe contributed significantly to the COVID-19 pandemic spreading throughout the world. BlueDot, based in Canada, applied machine learning and natural language processing to track, recognize, and report the spread of COVID-19, which they accomplished faster than the WHO or Centre for Disease Control and Prevention (CDCP) in the United States of America. It is projected that this technology, which is based on machine learning and natural language processing, can be leveraged in the future to predict zoonotic infection risk to humans using climate and human activities as variables. The prediction of individual risk profiles using the data extracted from social media such as family history and lifestyle as well as clinical, personal, and travel data can provide precise and accurate predictions. However, such technology can trigger privacy concerns [55]. Similarly, virtual healthcare assistant is a multilingual healthcare agent that has been developed based on natural language processing. It is a question–answering system that responds to questions related to COVID-19; it delivers trustworthy information on COVID-19 guidelines, protection measures, symptom monitoring and checking, and provides advice to individuals on their need for screening in the hospital or self-isolation. The virtual healthcare assistant was developed by a Canada-based organization [55].

RETRACTED

### 5.4. Case Study: United States of America

In the United States, many medical centres are modifying their existing intelligent systems that were purposely meant to predict patients' illnesses. These intelligent systems are now being modified to predict specific types of COVID-19 outcomes, like the need for intubation. The intelligent systems are trained to learn the illness patterns by feeding the system with thousands of patient records as training data. However, there is insufficient data to build an entirely new intelligent system for predicting COVID-19. Therefore, researchers are assessing the existing tools with the aim of customizing them to help in the fight against the COVID-19 pandemic [20].

## 6. Conclusions

This paper proposes a solution framework based on machine learning for integration of the fight against COVID-19 in smart cities, from different viewpoints such as predicting COVID-19 vaccine immunogenicity, detecting COVID-19 severity, predicting COVID-19 mortality, COVID-19 resource allocation, COVID-19 drug discovery, COVID-19 contact tracing, detecting social distancing and wearing of masks, triage of COVID-19 patients, identifying COVID-19 patients requiring a ventilator, and predicting which COVID-19 patients might be beyond medical intervention. The paper presented a comprehensive guide for implementing the machine learning framework in smart cities. The solution framework can potentially automate the means of fighting the COVID-19 pandemic in smart cities from multiple dimensions. This would ease the fatigue of the healthcare workers due to the very high number of COVID-19 patients requiring medical attention simultaneously and provide widespread access to a quality healthcare system. In addition, this study foresees that the proposed smart city machine learning-based framework used in combatting COVID-19 will be an essential guide for the research community in developing more compartmentalized forecasting and analyzing tools, with the prospect of mitigating the spread of the COVID-19 pandemic and the occurrences of any similar future disease pandemics. The limitation of the study is inherent in the pieces of the framework being still in their design form and so not yet pieced together in implementation form. However, as seen in several studies, components of the framework have already been implemented, which confirms its applicability. In future work, it will be interesting to see the real-world application of the proposed framework and further investigate the practicality of the model and its efficiency in smart city environments. This deployment of the proposed framework should generate policies to allow for effective integration into the city's existing social and health systems.

RETRACTED

## Figures and Tables

**Figure 1:** Proposed smart city framework integrated with machine learning for fighting COVID-19.

**Figure 2:** Typical transfer learning model for predicting future pandemics.

**Figure 3:** Application and flow of machine learning and other subdomains of AI in combatting COVID-19.

**Table 1:** Summary of the application of machine learning in drugs discovery.

Reference	Study approach	Advantage	Challenge
[67]	Deep learning-based computational drug discovery	The generated molecules could serve as a good drug potential for SARS CoV and COVID-19. The results also show that a deep learning model is important in testing the current compound and obtaining a new molecule for use in COVID-19 drugs	By utilizing limited data for model training, there could be a degree of error due to inaccuracies in parameter values
[68]	Target-specific and selective drug design for COVID-19 using a deep generative model	The framework can take care of candidate generations for multiple targets by employing trained mode. Besides, it can also permit explicit accounting for offtarget selectivity	Large scale data size is required for an effective study
